# Virtual Reality and Cardiac Diseases: A Systematic Review of Applications and Effects

**DOI:** 10.1155/2023/8171057

**Published:** 2023-05-30

**Authors:** Hamid Bouraghi, Ali Mohammadpour, Taleb Khodaveisi, Marjan Ghazisaeedi, Soheila Saeedi, Sahar Familgarosian

**Affiliations:** ^1^Department of Health Information Technology, School of Allied Medical Sciences, Hamadan University of Medical Sciences, Hamadan, Iran; ^2^Department of Health Information Management and Medical Informatics, School of Allied Medical Sciences, Tehran University of Medical Sciences, Tehran, Iran; ^3^Clinical Research Development Unit of Farshchian Hospital, Hamadan University of Medical Sciences, Hamadan, Iran; ^4^School of Medicine, Hamadan University of Medical Sciences, Hamadan, Iran

## Abstract

**Introduction:**

Cardiac diseases have grown significantly in recent years, causing many deaths globally. Cardiac diseases can impose a significant economic burden on societies. The development of virtual reality technology has attracted the attention of many researchers in recent years. This study aimed to investigate the applications and effects of virtual reality (VR) technology on cardiac diseases.

**Methods:**

A comprehensive search was carried out in four databases, including Scopus, Medline (through PubMed), Web of Science, and IEEE Xplore to identify related articles published until May 25, 2022. Preferred Reporting Items for Systematic Reviews and Meta-Analyzes (PRISMA) guideline for systematic reviews was followed. All randomized trials that investigated the effects of virtual reality on cardiac diseases were included in this systematic review.

**Results:**

Twenty-six studies were included in this systematic review. The results illustrated that virtual reality applications in cardiac diseases can be classified in three categories of physical rehabilitation, psychological rehabilitation, and education/training. This study revealed that the use of virtual reality in psychological and physical rehabilitation can reduce stress, emotional tension, Hospital Anxiety and Depression Scale (HADS) total score, anxiety, depression, pain, systolic blood pressure, and length of hospitalization. Finally, the use of virtual reality in education/training can enhance technical performance, increase the speed of procedures, and improve the user's skills, level of knowledge, and self-confidence as well as facilitate learning. Also, the most limitations mentioned in the studies included small sample size and lack of or short duration of follow-up.

**Conclusions:**

The results showed that the positive effects of using virtual reality in cardiac diseases are much more than its negative effects. Considering that the most limitations mentioned in the studies were the small sample size and short duration of follow-up, it is necessary to conduct studies with adequate methodological quality to report their effects in the short term and long term.

## 1. Introduction

According to the Global Burden of Disease (GBD) 2017, cardiovascular diseases are estimated to cause 17.8 million deaths worldwide. 330 million years of life have been lost to this disease, and 35.6 million years have been lost to disability. Studies show that the most deaths among noncommunicable diseases are caused by cardiovascular diseases, which are the main cause of premature death worldwide [1]. These diseases impose a significant economic burden on societies and families and can have a negative impact on people's quality of life [2].

In the last decade, various technologies such as artificial intelligence, Internet of things, wearable smart sensors, mobile health, telemedicine, 3D printing, digital games, and others have been used in education, rehabilitation, diagnosis, prediction, and treatment of diseases [3–5]. The mentioned technologies can have positive effects on cardiovascular diseases. A systematic review study that investigated the effects of telecardiology has concluded that this technology has positive effects on early diagnosis, early treatment, mortality reduction, health care costs reduction, patient quality of life, and patient satisfaction [6]. In recent years, advanced technologies have made user-friendly interfaces feasible, and high-performance computers have made it possible to develop interactive virtual environments [7]. Virtual reality is one of the advanced technologies introduced in this regard. Virtual reality technology provides an all-around experience for users by simulating real-world scenarios and creating an interactive virtual environment using hardware and software facilities [8].

The term “virtual reality” is attributed to Jaron Lanier [9]. Virtual reality is defined as a technology that enables users to experience the sense of real-world without actually being in it. A key feature of virtual reality is the ability to create a virtual world for users. This allows the possibility of creating a sense of immersion with the help of equipment such as headphones and virtual reality headsets. In addition, there is the possibility of providing sensory feedback and the possibility of interaction between the user and the virtual world. Virtual reality has been used in various medical fields, including physical rehabilitation, cognitive rehabilitation, education, and pain reduction [10–13]. The mentioned technology can be used in both chronic diseases and infectious diseases [14–18].

Various studies have confirmed the positive effects of virtual reality on psychiatric disorders, physical rehabilitation, and education. In psychiatric disorders, evidence shows that VR can reduce pain, anxiety/phobias, post-traumatic stress disorder, fear of driving or flying, agoraphobia, claustrophobia, and arachnophobia [19]. In physical rehabilitation, evidence shows the positive effect of VR on upper limb function but does not show any effect on gait, hand agility, and balance [20]. Also, in education, VR can increase the postintervention knowledge of health care professionals and improve skill outcomes [21].

This cutting-edge technology can have various applications in cardiac diseases and offer different effects according to those applications. This technology can have various applications in cardiovascular diseases, including simulating heart surgery, practicing in specific circumstances before surgery, checking the proper status of the inner and outer heart wall layers, interacting with heart data and information with no physical touch by surgeons, rehabilitating patients after heart surgery, teaching heart anatomy to students, teaching cardiopulmonary resuscitation, and using this technology to reduce stress before surgery [22]. Before employing this technology in the field of cardiac diseases, it is essential to determine its effectiveness. By identifying the effectiveness of virtual reality, it can be suggested to patients and physicians, and by identifying its ineffectiveness, it is possible to avoid spending money and time.

This study aimed to provide an overview of the applications and effectiveness of virtual reality in cardiac diseases. We seek to identify the following:

1. What applications can virtual reality have in cardiac diseases?
2. Can this technology have positive effects on cardiac diseases?
3. What negative effects can virtual reality have in this area?
4. Which groups are the main users of virtual reality?
5. What limitations did the selected studies encounter in terms of VR applications?

## 2. Material and Methods

Preferred Reporting Items for Systematic Reviews and Meta-Analyzes (PRISMA) guideline was used to report how to conduct this systematic review and present its results [23].

### 2.1. Search Strategy

Four databases, including Scopus, Medline (through PubMed), Web of Science, and IEEE Xplore, were searched to investigate virtual reality's applications and effectiveness in cardiac diseases. No time limit was applied to the search for articles. Papers that were published until May 25, 2022, were included in the review. Key words such as virtual reality and cardiac disease and MeSH terms related to them were combined and used for the search. The search strategy related to the PubMed database is presented in Table 1. In order to search each of the databases, a search strategy was adapted according to that database, and then the search was carried out. No restrictions were applied to the search in the PubMed and Web of Science databases, but in the Scopus database, the search was limited to “article” and “conference paper” in terms of document type. In the IEEE Xplore database, only documents that were in the three categories of “conferences,” “journals,” and “early access articles” were included in the review.

### 2.2. Study Selection

In the search phase, no restrictions were applied (except for the document type in Scopus and IEEE Xplore databases), but inclusion and exclusion criteria were considered in reviewing the title and abstract of the articles, which are shown in Table 2.

### 2.3. Quality Assessment

The Effective Public Health Practice Project (EPHPP) was used to assess the quality of selected articles' methodology. With the help of this tool, the following six aspects can be examined:

1. Study design
2. Withdrawals and dropouts
3. Data collection practices
4. Selection bias
5. Blinding as part of a controlled trial
6. Confounders

This checklist can be used to assess the quality of quantitative studies. With the help of this tool and based on the previous criteria, studies can be classified as weak, moderate, and strong. The scoring of studies in the three categories is as follows:

1. Strong (no weak ratings)
2. Moderate (one weak rating)
3. Weak (two or more weak ratings)

The quality assessment of the selected articles was carried out by two authors. After completing the quality assessment, the results were compared by the two authors, and any disagreement was resolved through discussion with HB.

### 2.4. Data Extraction

In the first stage, the titles and abstracts of all retrieved articles were independently reviewed by two authors. Then, the full text of articles that seemed relevant was retrieved and analyzed, and the desired information was extracted from them. Also, the references of all articles were checked to find relevant articles. Any disagreement between the authors was resolved through discussion with HB. In order to extract the desired information from the articles, an Excel sheet was designed. The following information was extracted from the articles and entered into the Excel spreadsheet: study, author name, type of publication (journal or conference paper), journal or conference name, year, country, target group, type of VR application, intervention group/control group, detail of groups (sex, age), sample size, session detail, measured outcome, results in VR condition, study limitations, and outcome.

Also, an Excel sheet was designed to assess the quality of articles based on quality assessment criteria.

### 2.5. Data Analysis

Due to the diversity that exists in the application of virtual reality in cardiac diseases as well as the diversity in its effects, a meta-analysis was not performed, and a narrative synthesis was used to report the results.

## 3. Results

### 3.1. Results of the Literature Search

The process and results of the search and selection of articles based on the PRISMA diagram are shown in Figure 1. The search in four databases (Scopus, ISI Web of Science, Medline (via PubMed), and IEEE Xplore) resulted in the retrieval of 4848 articles. After removing duplicates, 3,348 articles remained, and their title and abstract were examined. By reviewing the title and abstract, 3,315 articles were unrelated or did not meet the inclusion criteria. Finally, the full text of 33 articles was examined. A total of 26 studies that investigated the effects of virtual reality on cardiac diseases were included in this study, from which the desired items were extracted.  Figure 2 displays the word cloud of the included articles, which is a visual display of frequent keywords used in the title and abstract.

### 3.2. General Characteristics of the Included Studies

The general characteristics of the included studies are given in Table 3. Examining the trend of published studies shows that the use of VR in cardiac diseases has increased over the years, and the largest number of studies (*N* = 10, 38.5%) was related to the year 2021. The most recent study was published in 2022, while the oldest was published in 2005.

The continents and countries, in which the studies had been conducted, are shown in Figure 3. No studies had been conducted in the continents of Australia and Africa, and the continent of Europe accounted for the largest number of studies (*N* = 10, 38.5%). Poland, Brazil, and the USA had the most published studies, with four each. None of the published studies were conference papers, and all of them had been published in journals. Two journals, Archives of Physical Medicine and Rehabilitation and Journal of Medical Internet Research with two articles each, had published more articles related to VR in cardiac diseases than the other journals.

Three groups of people were the target users of the applied technology: (1) patients (*n* = 18, 69%), (2) students (*n* = 7, 27%) and (3) care providers (*n* = 1, 4%). VR applications can generally be classified into two categories of rehabilitation and education/training (Figure 4). The results of present study revealed that, the most use of VR was in rehabilitation with 17 studies. VR was also used in nine studies to train students. The minimum sample size of the included studies was 18 and the maximum was 180 (IQR1: 27, median: 34.5, IQR3: 60).

### 3.3. Effects of Virtual Reality on Cardiac Patients

Table 4 illustrates the effects of virtual reality applications on cardiac patients. The effects, according to the type of VR application, can be classified into two general categories, namely, rehabilitation (physical and psychological) and education/training.

#### 3.3.1. Effects of VR in Rehabilitation

The positive effects of VR in rehabilitation can be assessed in two general categories, namely, physical rehabilitation and psychological rehabilitation. For each of these rehabilitations, positive effects were reported in nine studies. The use of VR in physical rehabilitation had 22 positive effects, the most significant of which included reduction of pain and length of hospitalization, increase of METS (metabolic equivalents), and its positive effects on heart rate. In addition, this technology in psychological rehabilitation had 16 effects, including a reduction in stress, emotional tension, HADS total score, anxiety, and depression.

#### 3.3.2. Effects of VR in Education/Training

Among the positive effects of VR in education/training, we can point to improvements in technical performance, an increase in the speed of procedures, and improvements in the user's skills, level of knowledge, and self-confidence, as well as easier learning.

#### 3.3.3. Negative Effects of VR

Only in three studies (11.5%), the effects of VR were not positive. The VR group had lower satisfaction, engagement, and motivation than the control group in a psychological rehabilitation study. Also, in a study, the intervention group felt more pain than the control group. In regard to education/training, in only one study, technical skills, providing high-quality education, and delivering feedback were better in the control group than in the VR group.

### 3.4. Limitations Mentioned in the Studies

Fourteen limitations were mentioned in the examined studies (Table 5), the most important of which was “small sample size.” Also, the lack of follow-up or the short duration of follow-up was another limitation of the studies included in this systematic review.

### 3.5. Quality Assessment of the Included Studies

The results of the quality assessment of the reviewed articles are presented in Figure 5. According to the global rating score, 69% of the articles were assessed as strong. Only in terms of blinding, 81% of the studies were assessed as moderate, and in terms of other criteria, a higher percentage of studies were strong. Also, due to the fact that all the included studies were randomized trials, 100% of them were strong in terms of study design.

## 4. Discussion

This study was conducted to investigate the effectiveness of VR applications in cardiac diseases. For this purpose, a comprehensive search was conducted in four reliable databases. Finally, 26 studies that met the inclusion criteria were reviewed, and the desired information was extracted from them. The results of this review revealed that most studies had been conducted in Europe (38.5%). We could classify the applications of VR into two general categories, namely, rehabilitation and education/training. Users of this technology in the abovementioned areas include patients, students, and health care providers. This technology has been shown to have many positive effects on physical rehabilitation. These include a reduction in pain and length of hospitalization, an increase in METS, and its positive effects on heart rate. In psychological rehabilitation, these effects include a reduction in stress level, emotional tension, HADS total score, anxiety, and depression. Also, in training/education, the positive effects of VR include improvements in technical performance, an increase in the speed of procedures, and improvements in the user's skills, level of knowledge, and self-confidence, as well as easier learning.

According to the findings of this study, the use of virtual reality in cardiac patients can also result in pain reduction. Various studies are in line with the present study in demonstrating the positive effects of VR on pain reduction. A systematic review conducted by Iannicelli and colleagues [49] for pediatric patients concluded that VR is a practical tool for nonpharmacological reduction of pain. Also, a systematic review conducted by Smith and colleagues on the role of VR in pain management in inpatient settings revealed that 67% of the included studies reported a significant reduction in pain [50]. Also, other studies have shown the effectiveness of VR in reducing pain in cancer, ankylosing spondylitis, and postmastectomy patients, as well as neuropathic pain in spinal cord injuries [51–53]. Based on the previous studies, virtual reality has significant potential for reducing pain. It can also be used in cardiac patients, especially after surgery.

One of the applications of VR in cardiac diseases is for education/training. The most significant effects of VR in education/training include improvements in technical performance, an increase in the speed of procedures, and improvements in the user's skills, level of knowledge, and self-confidence, as well as easier learning. A systematic review by Choi and colleagues revealed the effectiveness of this technology in nursing education [54]. The results of a systematic review and meta-analysis that investigated the impact of virtual reality on health-related education revealed that virtual reality slightly improved the knowledge and cognitive skills of health care professionals in comparison to traditional learning [21]. The results of a study aimed at comparing the difference between training with virtual reality and other forms of simulation training showed no significant difference in the effectiveness of these two methods in endoscopy, which is contrary to the results of the present study [55]. Considering the increasing use of VR in education/training and the effectiveness of this technology in cardiac diseases, this technology can be used as a complementary training/education tool in complex processes in cardiac diseases such as cardiac catheterization or coronary artery bypass grafting.

Other benefits of virtual reality for cardiac patients include its psychological effects, including reducing stress levels, emotional tension, anxiety, and depression. A systematic review study in this field showed that virtual reality can reduce fatigue, tension, and depression and also lead to calmness and increased quality of life [56]. In another study, this technology had a positive effect on phobias [57]. Another study showed the positive effects of virtual reality on phobia and post-traumatic stress disorder [58]. Considering the positive effects of VR, especially in psychological rehabilitation, this technology can be used to reduce stress in cardiac patients before angiography, angioplasty, or surgery. Also, this technology can be used to reduce depression after coronary artery bypass grafting.

Although it can be said that virtual reality technology has been widely welcomed in some countries, in some parts of the world, such as the African continent, this technology has not yet been used broadly in healthcare. In recent years, another emerging technology called “metaverse,” which is a combination of several powerful technologies such as virtual reality, artificial intelligence, augmented reality, Internet of medical devices, quantum computing, and robotics [59, 60], has entered healthcare and can have various applications in the future in this field. It is recommended that these emerging technologies be applied in different countries and areas of health care and their effectiveness be reported.

With all the advantages mentioned for virtual reality, implementing this technology may face challenges and complications. One challenge that should be considered is the scalability of this novel technology. The important solution to this challenge is to have the right number of headsets to the right locations or provide alternative access options to learners. These alternative access options include desktop, routinely accessed through a URL, and mobile, which are available via a tablet or adaptable phone. Another solution is to use software such as an extended reality system (XRS) and the WebXR Device API. Another challenge that the use of virtual reality may have in health care is cybersickness, which should be considered before using this technology.

This study had several strengths and limitations. One of the strengths of this study was the comprehensive search in four valid databases to identify all related studies without time restriction. Reviewing the references of related studies to avoid missing relevant studies and evaluating the quality of articles were other strengths of this study. The limitation of this study was the exclusion of non-English studies.

## 5. Conclusion

This systematic review classified the applications of virtual reality in cardiac diseases into three categories, namely, physical rehabilitation, psychiatric rehabilitation, and education/training. The results of this systematic review showed that VR can have many positive effects on rehabilitation and training/education including reduction of pain and length of hospitalization, stress levels, emotional tension, anxiety, and depression and improvement in technical performance. Despite the various advantages mentioned for the use of virtual reality in cardiac diseases, the use of this technology is not without problems. For further studies, it is recommended that this technology be used with a larger sample size over a longer period and its effects be reported.

## Figures and Tables

**Figure 1:** Flow diagram of the literature search and study selection.

**Figure 2:** Word cloud of core keywords used in included papers.

**Figure 3:** The distribution of studies based on countries and continents.

**Figure 4:** Applications of virtual reality in cardiac diseases.

**Figure 5:** Quality assessment of the included studies.

**Table 1:** Keywords related to searching databases.

Keywords used for technology	Keywords used for disease
(“Virtual reality” (MeSH) OR “virtual realities”)	(“Cardiovascular diseases” (MeSH) OR “cardiovascular disease” OR “CVD” OR cardiovascular OR “circulatory system” OR “circulatory systems” OR circulatory OR heart (MeSH) OR hearts OR cardiac OR myocardium (MeSH) OR myocardia OR “myocardial infarction” (MeSH) OR “heart attack” OR “myocardial ischemia” OR “atrial fibrillation” OR atherosclerosis OR “peripheral artery disease” OR “coronary artery disease” OR “coronary heart disease” OR CHD OR MI OR “ischemic cardiovascular disease” OR ICD OR cardiomyopathy OR “heart disease” OR “heart arrest” OR “cardiac arrest” OR “angina” OR “vascular disease” OR CAD OR hypertension)

Search strategy: (keywords used for technology) AND (keywords used for disease).

**Table 2:** Inclusion and exclusion criteria for selecting articles.

Inclusion criteria	Exclusion criteria
(1) Studies in the English language (2) Virtual reality as a technology used in cardiac diseases (3) Articles that have reported the effectiveness (4) Randomized studies (5) Effects related to virtual reality were compared in the control and intervention groups	(1) Studies that investigated the effect of an intervention other than virtual reality (2) Studies that did not report the effectiveness of the mentioned technology (3) Letters to editors, review articles, protocols, monographs, and theses/dissertations (4) Articles whose full text was not in English

**Table 3:** General characteristics of included studies.

Author, year	Country	Journal	Target group	Type of VR application	Intervention group/control group	Sample size	Detail of groups (sex, age)	Session detail	Measured outcome	Outcome
Jozwik et al., 2022 [24]	Poland	Healthcare	Patients with CHD	Psychological rehabilitation	CR + VR vs CR + schultz autogenic training	*N* = 34 VR+ CR = 11 CG = 23	Sex: 34 M Age CG: 62.52 ± 7.18 EG: 66.55 ± 9.63	2 times a week for 4 weeks	(i) Anxiety level (ii) Depression level (iii) Emotional tension level (iv) External stress level (v) Intrapsychic stress level (vi) Risk of lying	This study verified that VR leads to an improvement in the mental state of the patients

Szczepanska-Gierachaet al., 2021 [25]	Poland	Cyberpsychology, behavior, and social networking	Patients with CAD	Psychological rehabilitation	CR + VR vs CR + schultz autogenic training	*N* = 32 VR+ CR = 15 CG = 17	Sex EG: 9 F, 6 M CG: 11 F, 6 M Age CG: 68.41 ± 5.06 EG: 69.47 ± 7.54	2 times a week for 4 weeks	(i) Anxiety level (ii) Depression level (iii) Emotional tension level (iv) External stress level (v) Intrapsychic stress level (vi) Risk of lying	This study confirmed that VR leads to an improvement in the mental state of the patients

Ribeiro et al., 2021 [26]	Brazil	Physiotherapy research international	Patients undergoing CABG	Physical rehabilitation	VR vs control group and EMG	*N* = 48 VR = 17 EMG = 15 CG = 16	Sex CG: 4 F, 11 M EMG: 2 F, 13 M VR: 7 F, 10 M Age CG: 60.3 ± 8.3 EMG: 58.3 ± 7.7 VR: 62.1 ± 9.0	Not clear	(i) Heart rate variability (ii) Time of discharge of hospital	Physiotherapy protocols, combined with VR training, improved a higher number of indicator indices and a shorter hospital stay after surgery

Patel et al., 2021 [27]	USA	The international journal of cardiovascular imaging	Medical students, residents, fellows, nurses, advanced practitioners, junior attending physicians, dieticians, and bioengineering PhD students	Anatomy education	VR vs a desktop computer interface	*N* = 51 VR = 24 CG = 27	Sex CG: 18 F, 9 M VR: 16 F, 8 M Age CG: 30 VR: 28	Not mentioned	(i) Visuospatial knowledge	There was no statistically significant difference between VR and the control group

Laghlam et al., 2021 [28]	France	Annals of intensive care	Patients undergoing cardiac surgery	Psychological rehabilitation	VR vs kalinox	*N* = 180 VR: 90 CG90	Sex CG: 18 F, 72 M VR: 28 F, 62 M Age CG: 68 VR: 68	5 min before the removal of the drains, and was continued for 10 min after	(i) Pain level (ii) Anxiety level	Although VR was well tolerated by patients and allowed a satisfying self-reported anxiety control, it failed to confirm noninferiority compared to Kalinox® for controlling pain and anxiety

Keshvari et al., 2021 [16]	Iran	Egyptian heart journal	Patients undergoing coronary angiography	Physical rehabilitation/psychological rehabilitation	VR vs usual care	*N* = 80 VR = 40 CG = 40	Sex CG: 15 F, 25 M VR: 8 F, 32 M Age CG: 52.08 ± 4.002 VR: 50.95 ± 4.120	5 min for each patient	(i) Anxiety level (ii) Heart rate (iii) Respiratory rate (iv) Blood pressure	VR distraction was effective in reducing anxiety before coronary artery angiography

Jozwik et al., 2021 [29]	Poland	Journal of clinical medicine	Patients with CAD	Psychological rehabilitation	CR + VR vs CR + schultz autogenic training	*N* = 77 VR = 28 CG = 49	Sex CG: 25 F, 24 M VR: 17 F, 11 M Age CG: 63.96 ± 6.89 VR: 66.00 ± 9.73	8 sessions, 3 times a week	(i) Anxiety level (ii) Depression level (iii) General stress level (iv) Emotional tension level (v) External stress level (vi) Intrapsychic stress level	The virtual environment with standard CR leads to a significant improvement in patients' mental health

Jozwik et al., 2021 [30]	Poland	Medicina	Patients with IHD	Psychological rehabilitation	CR + VR vs CR + schultz autogenic training	*N* = 43 VR+ CR = 17 CG = 26	Sex CG: 26 F VR: 17 F Age CG: 65.23 ± 6.49 VR: 65.65 ± 10.07	3 times a week for 8 weeks	(i) Generalized stress level (ii) Emotional tension level (iii) External stress level (iv) Intrapsychic stress level (v) Depression level (vi) Anxiety level	VR therapy is an efficient and interesting supplement to cardiac rehabilitation, with proven efficacy in reducing stress levels

Gulick et al., 2021 [31]	USA	Journal of medical internet research	Patients undergoing cardiac rehabilitation	Physical rehabilitation/psychological rehabilitation	VR vs standard care	*N* = 35 VR = 16 CG = 19	Age: 61 ± 9.9	Not clear	(i) Knowledge retention (ii) Patient satisfaction (iii) Engagement	No improvements were seen in the VR group

da Cruz et al., 2021 [32]	Brazil	Physical therapy & rehabilitation journal	Patients with cardiovascular diseases or risk factors	Psychological rehabilitation	CR + VR vs traditional CR	*N* = 61 VR+ CR = 30 CG = 31	Sex CG: 7 F, 24 M VR: 15 F, 15 M Age CG: 66.83 ± 10.93 VR: 63.27 ± 12.68	3 times a week for 12 weeks	(i) Adherence (ii) Motivation (iii) Engagement	Although VR increased program adherence but decreased patient motivation and absorption

Chang et al., 2021 [33]	Taiwan	Journal of the Chinese medical association	AF patients preparing for ablation	AF preprocedural education	VR vs paper-based materials	*N* = 33 VR = 11 CG = 22	Sex CG: 8 F, 14 M VR: 9 F, 2 M Age CG: 30–40 (2), 40–50 (4), 50–60 (4), and >60 yrs (12) VR: 30–40 (0), 40–50 (1), 50–60 (4), and >60 yrs (6)	Not clear	(i) Self-efficacy (ii) Satisfaction	VR decreased periprocedural anxiety and smoothed the procedure of AF catheter ablation

Zinchenko et al., 2020 [34]	Russia	New ideas in psychology	Humanitarian students	Anatomy education	VR vs paper and 3D interactive model on a computer display	*N* = 45	Sex CG1: 9 M CG2: 8 M VR: 9 M Age CG1: 21.2 ± 2.3 CG2: 22.9 ± 3.5 VR: 22.7 ± 3.6	15 min	(i) Number of correct answers	VR was more efficient than reading texts or interacting with a 3D model on a computer screen

Katz et al., 2020 [35]	USA	Journal of medical internet research	Anesthesiology residents	ACLS training	VR vs high-fidelity simulation	*N* = 23 VR = 11 CG = 12	Sex: 17 M, 8 F Age: 25–35	Not clear	(i) Technical skills (ii) Behavioral skills (iii) Cost	Utilization of a VR-based team leader refresher for ACLS skills is comparable with HFS in several areas, including learner satisfaction

Hessabi, 2020 [36]	Iran	International journal of pharmaceutical and phytopharmacological research	Patients admitted to the CCUs	Psychological rehabilitation	VR vs usual care	*N* = 60 VR = 30 CG = 30	Sex CG: 15 M, 15 F VR: 15 M, 15 F Age CG: 49.92 ± 7 VR: 52.03 ± 6	On the second and third night of admission for 15 min	(i) Anxiety level	VR can effectively reduce anxiety in hospitalized patients in the CCU

García-Bravo et al., 2020 [37]	Spain	International journal of environmental research and public health	Patients with IHD	Physical rehabilitation/psychological rehabilitation	CR + VR vs traditional CR	*N* = 20 VR = 10 CG = 10	Age CG: 53.7 ± 10.30 EG: 48.70 ± 6.66	2 times a week for 8 weeks (60 min)	(i) Ergometry (ii) Metabolic equivalents (iii) Functional independence measure (iv) 6MWT (v) Aerobic capacity and endurance (vi) Quality of life (vii) Depression level (viii) Satisfaction (ix) Adherence	VR could be incorporated into CR programs

Alves da Cruz et al., 2020 [38]	Brazil	Archives of physical medicine and rehabilitation	Patients with cardiovascular diseases or risk factors	Physical rehabilitation	VR vs regular CR	*N* = 27	Sex: 14 M, 13 F Age: 63.40 ± 12.71	Each VRBT or CR session lasted 85 minutes	(i) Heart rate (ii) Blood pressure (iii) Respiratory rate (iv) Rating of perceived exertion (v) peripheral oxygen saturation (vi) Heart rate reserve (vii) How long the patient maintained the prescribed (viii) HRR	VR produces similar physiological acute hemodynamic effects in CR

Maresky et al., 2019 [39]	Canada	Clinical anatomy	Medical students	Anatomy education	VR vs independent study	*N* = 42 VR = 28 CG = 14	Age: 18–34	30 min	(i) Number of correct answers	This study demonstrates the viability and the effectiveness of VR in teaching cardiac anatomy

Vieira et al., 2018 [40]	Portugal	Disability and rehabilitation: assistive technology	Patients with CAD	Physical rehabilitation/psychological rehabilitation	VR vs usual care and paper booklet	*N* = 33 VR = 11 EG2 = 11 CG = 11	Sex: 33 M Age EG1: 55 ± 9.0 EG2: 59 ± 11.3 CG: 59 ± 5.8	3 times a week for 6 months	(i) Executive function (ii) Ability to switch information (iii) Working memory (iv) Selective attention (v) Conflict resolution ability (vi) Quality of life (vii) Depression level (viii) Anxiety level (ix) Stress level	The VR improved attention and conflict resolution ability, revealing the potential of CR, specifically with virtual reality exercise, on executive function

Vieira, 2017 [41]	Portugal	European journal of integrative medicine	Patients with CAD	Physical rehabilitation	VR vs usual care and paper booklet	*N* = 33 EG2 = 11 CG = 11	Sex: 33 M Age EG1: 55 ± 9.0 EG2: 59 ± 11.3 CG: 59 ± 5.8	3 times a week for 6 months	(i) Total cholesterol levels (ii) High-density lipoprotein (iii) Low-density lipoprotein (iv) Triglycerides (v) Lean mass (vi) Body mass index (vii) Body fat at the trunk (viii) Total body fat (ix) Waist-to-height ratio	VR had a positive effect on body composition

Voelker et al., 2016 [42]	Germany	Journal of interventional cardiology	Cardiology fellows	Cardiac catheterization training	VR vs lectures	*N* = 18 VR = 9 CG = 9	Not mentioned	7.5 hours	(i) Participant's performance quality (ii) Procedure time (iii) Fluoroscopy time	VR simulation training improved the performance level of cardiology fellows

Valdis et al., 2015 [43]	Canada	Innovations-technology and techniques in cardiothoracic and vascular surgery	Surgical trainees	Robotic cardiac surgery training	VR vs no training	*N* = 19 VR = 9 CG = 10	Sex CG: 6 M, 4 F VR: 8 M, 2 F Age CG: 29.9 ± 2.4 VR: 32.7 ± 6.1	The average duration of VR: 9.3 hours	(i) Standardized robotic internal thoracic artery harvest (ii) Mitral valve annuloplasty	VR can significantly improve the efficiency and quality of learning in robotic cardiac surgery

Khanal et al., 2014 [44]	USA	Journal of biomedical informatics	Care providers	ACLS training	VR vs traditional ACLS training	*N* = 148	Sex: 10 M, 138 F	30 minutes	(i) Time for each task	VR-based ACLS training can provide a learning experience similar to face-to-face training

Cacau et al., 2013 [45]	Brazil	Revista brasileira de cirurgia cardiovascular	Patients in the postoperative period	Physical rehabilitation/psychological rehabilitation	VR vs conventional physical therapy	*N* = 60 VR = 30 CG = 30	Sex CG: 16 M, 14 F VR: 13 M, 17 F Age CG: 52 ± 2.4 VR: 49.2 ± 2.6	Twice a day	(i) Functional performance (ii) 6MWT (iii) Length of hospitalization (iv) Functional independence measure (v) Quality of life	Adjunctive treatment with VR demonstrated better functional performance in patients

Bagai et al., 2012 [46]	Canada	Circulation-cardiovascular interventions	Cardiology trainees	Cardiac catheterization training	VR vs apprenticeship-based training	*N* = 27 VR = 11 CG = 15	Sex CG: 13 M, 2 F VR: 5 M, 6 F Age CG: 31 VR: 29	Not mentioned	(i) Mounting the catheter on the guidewire (ii) Cannulating the coronary arteries exchanging catheters (iii) Obtaining and interpreting standard angiographic views (iv) Overall assessment of wire catheter skills (v) Time, efficiency, and ability to complete the case (vi) Need for verbal prompts (vii) Attending take over	Skills required to perform cardiac catheterization can be learned via mentored simulation training

Chuang et al., 2006 [47]	Taiwan	Physical therapy	Patients undergoing CABG	Physical rehabilitation	VR vs usual rehabilitation	*N* = 20 VR = 10 CG = 10	Sex: 20 M Age CG: 63.70 ± 10.03 VR: 65.70 ± 14.48	2 times a week for about 3 months (30 min)	(i) Heart rate (ii) VO_2_max (iii) Treadmill grades and speeds (iv) Blood pressure	This study showed a powerful effect of VR on the progress of cardiac rehabilitation

Chuang et al., 2005 [48]	Taiwan	Archives of physical medicine and rehabilitation	Patients undergoing CABG	Physical rehabilitation	VR vs usual rehabilitation	*N* = 32 VR = 17 CG = 15	Sex CG: 13 M, 2 F VR: 15 M, 2 F Age CG: 68.67 ± 12.32 VR: 64.41 ± 7.66	2 times a week for about 3 months (30 min)	(i) Heart rate (ii) Blood pressure (iii) Rating of perceived exertion (iv) VO_2_max	Treadmill training enhanced by VR was superior to conventional exercise protocols for post-CABG patients

CHD: coronary heart disease; CR: cardiac rehabilitation; CG: control group; EG: experimental group; CAD: coronary artery disease; CABG: coronary artery bypass graft; EMG: early mobilization group; IHD: ischemic heart disease; AF: atrial fibrillation; ACLS: advanced cardiac life support; HFS: high-fidelity simulation; CCU: cardiac care unit; 6MWT: 6-minute walk test; VRBT: virtual reality-based therapy.

**Table 4:** Effects of virtual reality in patients with cardiac diseases.

Outcome category	Outcomes subcategory	Outcomes	Positive effect	No effect	Negative effect
Rehabilitation	Physical	↓ Pain	[26, 45]		
		↓ Length of hospitalization	[26, 45]		
		↑ METS (metabolic equivalents)	[37, 48]		
		↑ OR ↓ heart rate	[16, 38]		
		↑ Walking capacity	[45]		
		↑ Energy level	[45]		
		↑ Physical ability		[45]	
		↑ Executive function	[40]		
		↑ Respiratory rate	[38]		
		↑ Maximum workload	[47]		
		↑ Rating of perceived exertion	[38]		
		↓ Systolic blood pressure	[16]		
		↑ Parasympathetic activity	[26]		
		↑ Cardiac autonomic modulation	[26]		
		↑ 6MWT	[37]	[31]	
		↑ Ergometry	[37]		
		↓ Total fat	[41]		
		↓ Waist-to-hip ratio	[41]		
		↑ High-density lipoprotein cholesterol	[41]		
		↑ General health	[37]		
		↑ VO_2_ peak	[48]		
		↓ Number of sessions required to reach the target HR and VO_2_	[47]		
	Psychological	↓ Stress level	[24, 25, 29, 30]	[40]	
		↓ Emotional tension	[24, 25, 29, 30]	[45]	
		↓ HADS total score	[24, 25, 29, 30]		
		↓ Anxiety	[16, 24, 25, 36]	[28, 40]	
		↓ Depression	[25, 29, 30, 37]	[40]	
		↑ Quality of life		[40]	
		↑ Selective attention	[40]		
		↑ Conflict resolution ability	[40]		
		↓ Feeling of pain			[28]
		↑ Satisfaction	[37]	[31]	[28]
		↑ Adherence	[32]		
		↑ Engagement		[31]	[32]
		↑ Motivation			[32]
		↑ Knowledge retention		[31]	
		↑ Social function	[37]	[45]	
		↑ Vitality	[37]		
Training and education	ACLS training	↑ Performance	[44]		
		↑ Technical skill			[35]
		↑ Providing high-quality education			[35]
		↑ Delivering feedback			[35]
		↑ Easiness	[35]		
		↑ Cost-effective	[35]		
	AF preprocedural education	↑ Familiarity	[33]		
		↓ Anxiety	[33]		
		↑ Self-efficacy	[33]		
		↑ Confidence	[33]		
		↑ Post-procedure self-monitoring-related knowledge	[33]		
		↑ General satisfaction	[33]		
		↓ Pain	[33]		
		↓ Impatience	[33]		
	Anatomy education	↑ Understanding of cardiac anatomy	[27, 39]		
		↑ Enjoyment	[39]		
		↑ Level of knowledge	[34]	[27]	
		↑ Subjects' impression of the ease of use	[27]		
	Cardiac catheterization training	↑ Technical performance	[46]		
		↑ Global performance	[46]		
		↑ Skills score	[42]		
	Robotic cardiac surgery training	↑ Proficiency scores	[43]		
		↑ Speed of internal thoracic artery harvest	[43]		
		↑ Speed of mitral annuloplasty	[43]		

**Table 5:** Limitations of included studies.

#	Study limitation	References
1	Small sample size	[24, 25, 27, 30, 32, 33, 35, 37, 39–42, 44]
2	Lack of or short duration of follow-up	[16, 24, 29, 30, 37, 46, 48]
3	Risk of selection bias	[27, 35, 37, 39, 39, 40]
4	large number of dropouts	[24, 29–31, 48]
5	Lack of measure of all variables in the present study	[35, 38, 44, 46]
6	Generalizability limitation	[28, 32, 35, 37]
7	Using of nonvalidated measure tool	[25, 28, 37]
8	Single blinded or not blinded	[33, 48]
9	Single-center study	[28, 32]
10	Heterogeneity of groups	[27, 46]
11	The possibility of a negative impact of the confounders on the results	[26, 32]
12	Use of inappropriate VR device	[28]
13	Difficulty to monitor the adherence to the exercise program	[40]
14	Using of a subjective assessment tool	[42]

## Data Availability

All data generated or analyzed during this study are included within the article.
